# Analysis of Apparent Diffusion Coefficient Value and Dynamic Contrast-Enhanced Magnetic Resonance Imaging Parameters of Prostate Cancer Patients after Diagnosis and Treatment with Magnetic Resonance Imaging

**DOI:** 10.1155/2022/3111054

**Published:** 2022-06-23

**Authors:** Peng Gu

**Affiliations:** Department of Urology Surgery, General Hospital of the Yangtze River Shipping, Wuhan, 430014 Hubei, China

## Abstract

This research was aimed at exploring the changes in the apparent diffusion coefficient (ADC) and dynamic contrast-enhanced magnetic resonance imaging (DCE-MRI) parameters of prostate cancer (PCa) patients. Sixty PCa patients from the hospital were recruited as the research object, and dynamic contrast-enhanced magnetic resonance imaging (DCE-MRI) scans were performed to determine the shape, scope, and enhancement characteristics of prostate lesions and their relationship with surrounding tissues. The quantitative parameters of ADC and DCE-MRI were measured. There were 4 patients (6.67%) with a Gleason score of 6 and 15 patients (25%) with a 4 + 3 score. The ADC with Gleason = 6 is 0.81 ± 0.08 × 10^−3^ s/mm^2^, the ADC with Gleason = 3 + 4 is 0.74 ± 0.07 × 10^−3^ s/mm^2^, the ADC with Gleason = 4 + 3 is 0.73 ± 0.05 × 10^−3^ s/mm^2^, the ADC with Gleason = 9 is 0.65 ± 0.06 × 10^−3^ s/mm^2^, and the ADC with Gleason = 10 is 0.59 ± 0.07 × 10^−3^ s/mm^2^. As the Gleason score increased, the ADC decreased and the permeation parameter transfer constant increased. When the ADC was combined with the permeability parameter transfer constant, the AUC of Gleason = 6 points and Gleason = 7 points was greatly different (*P* < 0.05). The 95% CI of the ADC combined permeability parameter transport constant when Gleason = 6 points and Gleason = 7 points was 0.898-0.934, the sensitivity was 75.4%, and the specificity was 86.2%. The ADC value was negatively correlated with Gleason score. The ADC value combined with VTC value has good diagnostic performance in evaluating the invasion of PCa, which is very important for making treatment plan and evaluating prognosis.

## 1. Introduction

Prostate cancer (PCa) refers to an epithelial malignant tumor that occurs in the prostate [1]. In recent years, due to lifestyle changes, the popularization of early screening, and the improvement of the level of diagnosis, the incidence of PCa in China has gradually increased, the risk of disease has increased with age, and it has begun to show a “younger” trend [2]. According to data from the National Cancer Center, PCa has become the most common malignant tumor in the male urinary system since 2008, and the incidence has continued to increase. In 2015, the morbidity rate reached 10.23/100,000, and the mortality rate was as high as 4.36/100,000 [3]. At present, the incidence of PCa in China has ranked 6th among men. In all patients with PCa, the early, middle, and late periods represent different treatment methods and different quality of life. The later it is discovered, the more difficult it will be to treat [4].

At present, the diagnostic methods of prostate cancer include prostate specific antigen and rectal index examination, but these methods cannot evaluate the invasion and pathological grade of the disease. The Gleason scoring system is the most commonly used method to evaluate the invasion of prostate cancer, and it has become one of the important reference indexes for clinical treatment plan and prognosis evaluation. Gleason score is an evaluation based on the fine running morphology of biopsy tissue under microscope. The scoring principle is that the score includes major structural types and minor structural types [5]. In recent years, more and more research results pointed out that multiparameter magnetic resonance imaging had good application prospects for the detection and classification of PCa. In particular, dynamic contrast enhanced magnetic resonance imaging (DCE-MRI) can be used for imaging evaluation of PCa. The intravenous bolus injection of contrast medium was used to evaluate the permeability of the tumor's microvessels and grade the malignant degree of the tumor [6]. Cybulski et al. [7] pointed out that there were differences in the volumetric metastasis constant between tumors of different grades, but when the tumor was located in the transition zone, there were most of the overlapping areas in the image. Due to the impact of the T2-weighted imaging projection effect, the diffusion coefficient cannot be detected in conventional magnetic resonance imaging, so apparent diffusion coefficient (ADC) was used to express the diffusion ability [8–11].

At present, most of the researches on the correlation between ADC value and quantitative parameters of DCE-MRI scan and prostate cancer at home and abroad are comparative studies between single-function imaging and pathological results, and most of them are retrospective studies. DCE-MRI was adopted to analyze the changes in ADC and DCE-MRI parameters of 60 prostate patients. This work is aimed at exploring the application value of DCE-MRI for PCa patients, which provided a reliable reference for clinical treatment.

## 2. Experimental Methods

### 2.1. Objects and Grouping

In this study, sixty male patients who were diagnosed with PCa in the hospital from January 2020 to November 2020 were recruited as the research objects. They underwent DCE-MRI scans and PCa biopsy under the guidance of rectal ultrasound. The average age was 62.47 ± 13.25 years old. This study had been approved by the ethics committee of the hospital, and all the subjects included in the study had signed the informed consent forms.

Inclusion criteria: (i) patients diagnosed with PCa and with a complete Gleason grading score, (ii) PCa treatment and needle biopsy were not performed before enrollment, and (iii) patients without contraindications for MRI scan.

Exclusion criteria: (i) the quality of the MRI image was poor, and severe artifacts can be seen; (ii) the urinary catheter can be found in the lesion in the MRI image; (iii) patients who had been treated in six months before enrollment; (iv) patients with severe allergies to the medication used; and (v) patients with abnormal blood coagulation function.

### 2.2. DCE-MRI Scanning

A superconducting magnetic resonance scanner was employed, with 8 channel body phase front coil, and DCE-MRI scanning was performed. Scanning parameters are shown in Table 1. The scan covered the entire prostate gland and the seminal vesicle. The patient's breathing was trained before the scan to try to avoid abdominal breathing. Three phase T1WI plain scans with a rotation angle of 3°6°9° were performed before the DCE-MRI scanning, and the other parameters were consistent with those of the DCE-MRI scanning parameters for the calculation of T1 values. A high-pressure syringe was used to inject gadodiamide at 0.25 mL/kg body mass through the dorsal vein, which was rinsed with 20 mL normal saline to ensure complete injection of the drug into the bloodstream. DCE-MRI was performed in 32 continuous scans with 52 layers in each phase, and the scanning time was 5 min.

### 2.3. Data Analysis

ADC measurement was as follows. The obtained DCE-MRI scan data was transmitted to GE through the workstation, and the ADC image was obtained after processing with GE Function software. The region of interest (ROI) was manually placed to determine the ADC of different lesion areas. The ROI was 25-45 mm^2^. Three measurements were taken on the upper, middle, and lower levels of the low signal on T2WI and the high signal on DCE-MRI, and the average value was taken. Bleeding, calcification, urethra, and blood vessels should be avoided during measurement, and the corresponding ADC was recorded.

The software for determining quantitative parameters of DCE-MRI automatically generated the permeability parameter volume transfer constant (VTC), rate constant (RC), and average, maximum, and minimum of extravascular extracellular volume fraction (EEVF) of all pixels in the ROI. Since the increase in PCa blood perfusion led to changes in vascular permeability, the distribution of hemodynamic parameter values was generally skewed, so 75% of each parameter value was adopted in this research.

### 2.4. Statistical Methods

SPSS 19.0 was employed for data statistics and analysis. Mean ± standard deviation (*x* ± *s*) was how measurement data were expressed, and percentage (%) was how count data were expressed. One-way analysis of variance was used to compare ADC, VTC, RC, and EEVF between different groups. ADC was combined with VTC value, and receiver operating characteristic (ROC) curve analysis was performed. The sensitivity and specificity were estimated, and the AUC values were compared between the groups with the area under the ROC curve. The result *P* < 0.05 indicated statistical significance.

## 3. Results

### 3.1. Gleason Grading Results

Figure 1 shows the proportion of Gleason scores in PCa patients. Among 60 patients with PCa confirmed by pathological diagnosis, 4 patients (6.67%) had a Gleason score of 6, 8 patients (13.33%) had a 3 + 4 score, 15 patients (25%) had 4 + 3 points, 21 patients (35%) had 8 points, 10 patients (16.67%) had a score of 9, and 2 patients (3.33%) had a score of 10.

### 3.2. ADC of Gleason Score Grading

Figure 2 shows the ADC comparison of Gleason scoring. As the Gleason score increased, the ADC showed a gradual downward trend.

The ADC with Gleason = 6 is 0.81 ± 0.08 × 10^−3^ s/mm^2^, the ADC with Gleason = 3 + 4 is 0.74 ± 0.07 × 10^−3^ s/mm^2^, the ADC with Gleason = 4 + 3 is 0.73 ± 0.05 × 10^−3^ s/mm^2^, the ADC with Gleason = 9 is 0.65 ± 0.06 × 10^−3^ s/mm^2^, and the ADC with Gleason = 10 is 0.59 ± 0.07 × 10^−3^ s/mm^2^.

Each group was compared in pairs, and it was found that Gleason = 3 + 4 points and Gleason = 4 + 3 points were not statistically significant (*P* > 0.05), while comparisons between the other groups were remarkable (*P* < 0.05).

### 3.3. Results of Prostate DCE-MRI Quantitative Parameters (VTC, RC, and EEVF) in Gleason Scoring

Figure 3 shows the comparison results of quantitative parameters of DCE-MRI. As the Gleason score continued to increase, the permeability parameter transfer constant (VTC) also gradually increased. The difference between Gleason = 3 + 4 points and Gleason = 4 + 3 points was not statistically considerable (*P* > 0.05). The other groups were compared in pairs, the difference between Gleason = 6 points and Gleason = 7 points was remarkable (*P* < 0.05), and the difference between Gleason = 7 points and Gleason = 8 points was also remarkable (*P* < 0.05). Comparisons of Gleason = 8 points or more showed no great difference (*P* > 0.05). The change trend of rate constant (RC) and extravascular extracellular volume fraction (EEVF) did not show a notable increase or decrease trend, and the difference was not considerable (*P* > 0.05).

### 3.4. ROC Curve of ADC Value Combined with VTC Value in PCa Gleason Grading

Figure 4 shows the ROC curve of MRI parameters in different Gleason grades of PCa. There was no remarkable difference in the comparison of the AUC using ADC value or VTC value alone (*P* > 0.05). When the ADC value was combined with the VTC value, the difference in AUC between Gleason = 6 points and Gleason = 7 points was remarkable (*P* < 0.05), and the difference in AUC between Gleason = 7 points and Gleason = 8 points was remarkable (*P* < 0.05), but there was no remarkable difference in AUC between Gleason = 8 points and Gleason = 9 points (*P* > 0.05).

Table 2 is the prediction of 95% CI, sensitivity, and specificity using ADC value combined with VTC value and different Gleason classification. For Gleason = 6 points and Gleason = 7 points, the 95% CI of ADC+VTC value was 0.898-0.934, the sensitivity was 75.4%, and the specificity was 86.2%. For Gleason = 7 points and Gleason = 8 points, the 95% CI of ADC+VTC value was 0.726-0.945, the sensitivity was 82.6%, and the specificity was 88.6%. For Gleason = 8 points and Gleason = 9 points, the 95% CI of ADC+VTC value was 0.758-0.832, the sensitivity was 76.7%, and the specificity was 83.9%.

### 3.5. PCa DCE-MRI Image Performance Characteristics

Figure 5 shows the PCa DCE-MRI image. On the T2 sequence, a low-signal nodule appeared in the surrounding area with a normal higher signal. The lesion was located in the peripheral zone of the prostate. On T2WI, it was mainly manifested as a single or multiple nodular low signal area in the peripheral zone of high signal and diffuse low signal shadow in the peripheral zone of the prostate on one side. The lesion was located in the central gland. On T2WI, there was an irregular low-intensity shadow in the central gland. The contrast between the lesion and the surrounding tissues was poor. The tumor was located inside the prostate, the outer edge of the prostate was intact, and the boundary with the surrounding venous plexus was clear. The lesion invaded the capsule and caused the capsule to thicken, local bulge, seminal vesicles were invaded, and low signal appeared in the seminal vesicles with high signal on T2WI.

### 3.6. Complications in PCa Patients

Figure 6 shows the occurrence of complications in PCa patients. It was found that the PCa patients in this study had the highest incidence of hematuria and hematuria after puncture. There were 43 patients (71.67%) with hematuria, 19 patients (31.67%) with bloody stools, 8 patients (13.33%) with urinary tract infections, 4 patients with sepsis (6.67%), and 2 patients with hematospermia (3.33%).

## 4. Discussion

The number of newly developed cases of prostate cancer in men is increasing gradually, so it is necessary to introduce more conservative treatment options as a substitute for the standard of care for prostate cancer. Before making a treatment plan, it is necessary to better predict the invasiveness of the disease. At present, the most commonly used D'Amico risk group divides prostate cancer into three groups: low risk, medium risk, and high risk, and the corresponding Gleason scores are 6, 7, and 8~10, respectively. However, studies have proved that prostate cancer patients with Gleason score of 9~10, which is also a high-risk grade of prostate, have a higher mortality rate than those with score of 8. The same Gleason score is 7, but it includes 3 + 4 points and 4 + 3 points. Patients with 3 + 4 points in these two categories tend to have a better prognosis [12].

In this study, there were 4 patients (6.67%) with Gleason score of 6 points, 8 patients (13.33%) with 3 + 4 points, and 15 patients (25%) with 4 + 3 points. There were 21 patients (35%) with 8 points, 10 patients (16.67%) with 9 points, and 2 patients (3.33%) with 10 points. Among them, Gleason = 6 points meant low risk, 7 points meant medium risk, and 8-10 points meant high risk. The ADC values of 60 PCa patients with different Gleason scores were analyzed, and the results showed that with the increase of Gleason score, the ADC showed a gradual decline trend [13]. Then, each group was compared in pairs, and it was found that Gleason = 3 + 4 points and Gleason = 4 + 3 points were significantly different (*P* > 0.05). The difference between the other groups was also remarkable (*P* < 0.05). It may be that the outer space between the cells was compressed, which limited the diffusion of water molecules, the MRI signal became higher, and the ADC value decreased. With the increase of PCa cell invasion, the adenoid structure gradually became solid and flaky [14, 15]. Ogura et al. [16] pointed out that the higher the degree of PCa malignancy, the lower the ADC value, which was consistent with the results of this study. Fukunaga et al. [17] pointed out that with the increase of Gleason score, ADC value tends to decrease, which is similar to the result of this study.

With the continuous increase of the Gleason score, the permeability parameter transport constant (VTC) in the quantitative parameters of DCE-MRI also gradually increased. The difference between Gleason = 3 + 4 points and Gleason = 4 + 3 points was not obvious (*P* > 0.05), but the difference between Gleason = 6 points and Gleason = 7 points was remarkable (*P* < 0.05). The difference between Gleason = 7 points and Gleason = 8 points was substantial (*P* < 0.05), which indicated that the differentiated PCa tissue had few atypia, slow cell metabolism, gradually reduced nutrient requirements, and lower tissue irrigation and capillary permeability. However, as the degree of deterioration of PCa cells deepened, tissue metabolism was vigorous, the demand for substances gradually increased, and the VTC value also increased [18].

When the ADC value was combined with the VTC value, the AUC difference between Gleason = 6 points and Gleason = 7 points was remarkable (*P* < 0.05), and the difference in AUC between Gleason = 7 points and Gleason = 8 points was also remarkable (*P* < 0.05). It showed that the ADC value combined with the VTC value had a good diagnostic performance, and the effect was ideal in terms of sensitivity [19, 20].

The disadvantage of this study is that the sample size of this study is small, which may be affected by the selection and verification bias. The number of samples in each grade is unevenly distributed. The moderate correlation or lack of correlation between MRI and histopathological parameters may also lead to its measurement error. For example, Gleason score is scored subjectively, and human factors such as experience will definitely play a role in reading accuracy.

## 5. Conclusion

DCE-MRI was performed to evaluate the ADC value and parameter changes of PCa patients. The ADC value was negatively correlated with Gleason score. The ADC value combined with VTC value has good diagnostic performance in evaluating the invasion of PCa, which is very important for making treatment plan and evaluating prognosis. In short, this study provides a good evidence-based basis for the clinical use of DCE-MRI to evaluate the data parameters of MRI of PCa patients.

## Figures and Tables

**Figure 1:** Proportion of Gleason score grades of PCa patients.

**Figure 2:** ADC comparison of Gleason score grading.

**Figure 3:** Comparison of quantitative parameters of DCE-MRI: (a) VTC; (b) RC; (c) EEVF. ^∗^Compared with Gleason = 7, *P* < 0.05.

**Figure 4:** ROC curves of MRI parameters in different Gleason grades of PCa. (a) Gleason = 6 points and Gleason = 7 points MRI parameter comparison ROC curve. (b) Gleason = 7 points and Gleason = 8 points MRI parameter comparison ROC curve. (c) Gleason = 6 points and Gleason = 7 points MRI parameter comparison ROC curve.

**Figure 5:** PCa DCE-MRI images. (a) A typical high signal had low signal shadow in the peripheral band, and the ADC value showed a low signal indicating that the dispersion was limited. (b) The normal central zone was clearly visible in the T2WI and ADC images, and the bilateral symmetry of the diffracted seminiferous duct was low signal. (c) PCa in the left central zone with surrounding tissues. (d) Left seminal vesicle gland involvement.

**Figure 6:** The occurrence of complications: (a) hematuria, (b) blood in the stool, (c) urinary tract infection, (d) sepsis, and (e) blood sperm.

**Table 1:** Scan parameters of DCE-MRI.

Items	Scanning parameters
Repeat time (ms)	3.8
Echo time (ms)	1.4
Flip degree	12°
Field of view (mm)	420-300
Layer thickness (mm)	5.0
Layer distance (mm)	-1.5
Whether to press fat	Yes
Matrix	256 × 192
*b* value (s·mm^−2^)	/
Number of incentives	0.73

**Table 2:** The prediction of 95% CI, sensitivity, and specificity using ADC value combined with VTC value and different Gleason classifications.

Gleason grade	95% CI	Sensitivity	Specificity
Gleason = 6 points and Gleason = 7 points			
ADC+VTC	0.898-0.934	0.754	0.862
Gleason = 7 points and Gleason = 8 points			
ADC+VTC	0.726-0.945	0.826	0.886
Gleason = 8 points and Gleason = 9 points			
ADC+VTC	0.758-0.832	0.767	0.839

## Data Availability

The data used to support the findings of this study are available from the corresponding author upon request.
